The article "(5E,7E)-4,5,6 Trihydroxy-3-(hydroxymethyl)tetrahydro-2H-pyran-2-ylheptadeca-5,7-dienoate from Euclea crispa (L.) Inhibits Ovarian Cancer Cell Growth by Controlling Apoptotic and Metastatic Signaling Mechanisms" was retracted in 2023. Reasons: signs of a paper mill; suspected computer-generated content; unreliable results or conclusions; concerns about the data.

# (5E,7E)-4,5,6 Trihydroxy-3-(hydroxymethyl)tetrahydro-2H-pyran-2-ylheptadeca-5,7-dienoate from *Euclea crispa* (L.) Inhibits Ovarian Cancer Cell Growth by Controlling Apoptotic and Metastatic Signaling Mechanisms

**DOI:** 10.1155/2022/4464056

**Published:** 2022-01-29

**Authors:** Chella Perumal Palanisamy, Bo Cui, Hongxia Zhang, Selvaraj Jayaraman, Ponnulakshmi Rajagopal, Vishnu Priya Veeraraghavan

**Affiliations:** ^1^State Key Laboratory of Biobased Material and Green Papermaking, College of Food Science and Engineering, Qilu University of Technology, Shandong Academy of Science, Jinan 250353, China; ^2^Centre of Molecular Medicine and Diagnostics (COMManD), Department of Biochemistry, Saveetha Dental College and Hospitals, Saveetha Institute of Medical and Technical Sciences, Saveetha University, Chennai 600 077, India; ^3^Central Research Laboratory, Meenakshi Academy of Higher Education and Research (Deemed to be University), Chennai 600 078, India

## Abstract

Bioactive compound (5E,7E)-4,5,6 trihydroxy-3-(hydroxymethyl)tetrahydro-2H-pyran-2-ylheptadeca-5,7-dienoate (compound 2) was isolated from *Euclea crispa* (*E. crispa*) by the chromatographic methods. Further, the compound was confirmed by spectroscopic techniques such as ultraviolet-visible (UV/Vis) spectrometer, Fourier transform infrared (FTIR) spectrometer, and ^1^H and ^13^C nuclear magnetic resonance (NMR). Compound 2 exhibited a significant antioxidant activity with IC_50_ values. It restrained the auxesis of HO-8910 cells in a shot-dependent mode. CXCR4, HER2, and Akt proteins involved in cell proliferation and metastasis were found to be significantly reduced (*p* < 0.05). The protein that is responsible for the death of cells (Bcl-2 and Bcl-xL) was reduced (*p* < 0.05), while the protein expression of p53 and caspase-9 was increased (*p* < 0.05) in compound 2-treated HO-8910 cells. The results of molecular docking analysis showed the binding affinity with CXCR4 and HER2. Thus, compound 2 can serve as a promising chemotherapeutic agent for the intervention of ovarian cancer. The findings of this study conclude that compound 2 from *E. crispa* might work as a potential antioxidative and chemotherapeutic agent. The *in vivo* studies and attempts will pave way for this compound to be an effective drug hereafter.

## 1. Introduction

Ovarian cancer (OC) is one of the frequently diagnosed cancers, and it is found that every year more than two hundred thousand women have been diagnosed with the disease, which comprises around two percent of the population [1]. A report by the World Cancer Fund International states that Fiji records the highest number of cases in contrary to China and a few regions of Africa record the lowest number of cases where only four women in a hundred thousand are prone to the disease. The deaths that are caused by this particular disease annually record about fifteen thousand [2]. In recent times, many therapies and medications have come in an existence for the treatment of OC, namely chemotherapy, laser therapy, radiotherapy, gene therapy, hyperthermia, and surgery [3]. Usually, a combination of treatments has been in practice to cure the disease. In particular, chemicals, amputation of diseased portions, and radiations are predominantly used to treat the tumour [4]. However, the scientific community recognized that these interventions have disadvantages and limitations. Consequently, there is an imperative medical need for breakthrough drugs that have a practical therapeutic impact on OC [5].

The article "(5E,7E)-4,5,6 Trihydroxy-3-(hydroxymethyl)tetrahydro-2H-pyran-2-ylheptadeca-5,7-dienoate from Euclea crispa (L.) Inhibits Ovarian Cancer Cell Growth by Controlling Apoptotic and Metastatic Signaling Mechanisms" was retracted in 2023. Reasons: signs of a paper mill; suspected computer-generated content; unreliable results or conclusions; concerns about the data.

Plants have a long history of use for the treatment of human diseases, particularly cancer, which is a lethal disease that causes deaths in individuals at a high rate [6–8]. Several medicinal plants have been reported to exhibit a variety of pharmacological and/or life functions such as antioxidant, antimicrobial, anti-inflammatory, anticancer, and antidiabetic, due to the presence of some active phytocompounds and compounds that possess aromatic hydroxylated rings [9–11]. The bioactive elements play an essential function in drug discovery programs in manufacturing medicine [12–14]. The plant-derived biomolecules are recognized as an attractive and promising approach and possess high value in biomedical research for the development of drugs against cancer [15]. Interestingly, in the recent past decades, a noteworthy collection of novel advanced medicines has been obtained from the medicinal plants with the last twenty years witnessing successful investigations on natural products in the field of anticancer drug research in most parts of the world [16,17].

*Euclea crispa* Linn. (*E. crispa*) is a shrub/small tree with a single stem and is commonly grown in S. Africa. *E. crispa* is called as blue guarri in English. It belongs to the family Ebenaceae [18]. The plants carry a dense canopy of simple leaves of dull green colour and a rigid, leathery lineament. The bark varies from grey to brown and is often covered with lichens [19]. The flowers are small, waxy, pendulous yellow to greenish-white. The corollas are bell-shaped and are deeply lobed. The plant leaves are filled with medicinal values and are traditionally used by indigenous people to treat various diseases such as gonorrhea and scabies, and the roots are used in treating diabetes and rheumatism. The fruits are edible. The antioxidant activity of *E. crispa* leaves is investigated using the ethanolic extracts of the leaves by isolating the bioactive compounds [6,20]. Thus, the bioactive compounds are isolated as an initiative to also extend the horizon to predict the chemotherapeutic activities of the plant to benefit mankind.

The article "(5E,7E)-4,5,6 Trihydroxy-3-(hydroxymethyl)tetrahydro-2H-pyran-2-ylheptadeca-5,7-dienoate from Euclea crispa (L.) Inhibits Ovarian Cancer Cell Growth by Controlling Apoptotic and Metastatic Signaling Mechanisms" was retracted in 2023. Reasons: signs of a paper mill; suspected computer-generated content; unreliable results or conclusions; concerns about the data.

## 2. Materials and Methods

### 2.1. Plant Collection

The leaves of *E. crispa* were collected from the campus of Qwaqwa, during April 2017. As a first step, the plants were identified by Prof. AOT Ashafa Department of Plant Sciences, Faculty of Natural and Agricultural Sciences, University of the Free State, Qwaqwa Campus [11]. Secondly, the leaves were rinsed in water to eliminate the dirt, contaminants, and foliar debris, and then, they were made dry with the exposure of air to deplete water and finally powdered. The powdered plant source was stored in an airtight container at four-degree Celsius for future use.

### 2.2. Extract Preparation

Extraction was prepared by soaking 500 g of the plant material in 2500 ml of ethanol in a flask. Then, the flask was placed on a shaker for about 72 hours at room temperature. Filtration was done using a Whatman No.1 filter paper, and then, it was dried using a rotary evaporator to obtain a concentrated extract and was stored at 4°C for later use.

### 2.3. Compound Isolation

The compound was isolated using thin-layer chromatography (TLC). To seclude the elements, the ethanolic leaf extracts were used. 15 g of the extract was fractionated on the TLC silica gel column followed by successful elusion using petroleum ether (3 × 30 cm), petroleum ether: chloroform (8 : 2, 6 : 4, 4 : 4, 2 : 8 v/v), and chloroform (100%), respectively. Then, the fractions were gathered in a 20 ml test tube and analyzed individually using TLC plates to affirm the presence of saturated fraction and confirmed by the appearance of a blot.

### 2.4. Structural Characterization

In a secluded compound, the presence of a functional group was identified using a Fourier transform infrared spectrometer with a resolution of 0.1/cm. To analyze the optical activity of compounds, the polarimetry technique was used and the instrument used was the PerkinElmer Polarimeter (Model 341). To investigate the purity of the sample, the NMR spectra were performed on the CDC13 solutions and the results were recorded on a Bruker DRX-500 NMR Spectrometer at 500 MHz, and the signals were considered as reference [21].

### 2.5. Antioxidant Activity

DPPH radical scavenging assay is the simplest mode to evaluate the antioxidant potential of a compound or extract. It is a unique method to carry out the reaction of the sample with DPPH in methanol/water, which facilitates in extracting the antioxidant compounds from the samples. DPPH radical scavenging assay was measured by the standard method [22]. The endothelial cells, macrophages, and neurons generate nitric oxide, which involves in the regulation of different physiological processes. Also, they serve as mandatory chemical mediators. Nitric oxide was generated by sodium nitroprusside (SNP) and measured [23]. Hydroxyl radical discarding activity of the isolated compound was measured according to Kunchandy and Rao [24]. The reducing power capacity was calculated by the modified method of Oyaizu [25]. Ferric reducing the power of the secluded compound was determined using the FRAP assay [26]. All tests were performed thrice.

The article "(5E,7E)-4,5,6 Trihydroxy-3-(hydroxymethyl)tetrahydro-2H-pyran-2-ylheptadeca-5,7-dienoate from Euclea crispa (L.) Inhibits Ovarian Cancer Cell Growth by Controlling Apoptotic and Metastatic Signaling Mechanisms" was retracted in 2023. Reasons: signs of a paper mill; suspected computer-generated content; unreliable results or conclusions; concerns about the data.

### 2.6. Computational Molecular Analysis

#### 2.6.1. Ligand Selection Preparation

The identified natural compounds and the FDA-approved drug (cyclophosphamide) were prepared using a default setting in LigPrep (LigPrep, Schrödinger, LLC, New York, NY, 2017).

#### 2.6.2. Protein Structure Preparation

The first step involved in the preparation of protein structure is retrieving the 3-dimensional (3D) structure of proteins from Protein Data Bank (PDB). The protein structures of CXCR4 and HER2 were obtained from the PDB (PDB IDs: 30E6 and 3BE1, respectively). Further, a grid-based ligand docking method was employed for protein preparation wizard with energetics.

#### 2.6.3. Active Site Prediction

Active site prediction is an important step since they play a crucial role in docking. The identified and characterized active sites and functional residues of the proteins of CXCR4 and HER2 were found using the software Sitemap. Grid points were used to characterize and identify proteins. The active sites in proteins may vary, and there may be one or more active binding sites where a ligand binds to the receptor. The active site and functional residues of CXCR4 and HER2 were recognized and qualified using Sitemap (SiteMap, Schrödinger, LLC, New York, NY, 2017). As an initial step, the Sitemap calculation gets started or characterized using the grid points through which the areas on the surface of the protein that was best suited for the ligands to bind were recognized. Sitemap highlights the regions with the binding site for occupancy by hydrophobic groups or by ligand hydrogen bond donors.

#### 2.6.4. Molecular Docking Analysis

All docking analysis was performed using the standard precision (SP), which is the standard mode of a grid-based ligand docking with energetics(Glide, Schrödinger, LLC, New York, NY, 2017). Docking was performed using Glide for the isolated natural compound and CXCR4 and HER2, and in the receptor grid generation, the van der Waals radius was 1.0. The force field used for the docking protocol was OPLS_2005. In the majority of the conformations, the lowest energy complexes were identified.

The article "(5E,7E)-4,5,6 Trihydroxy-3-(hydroxymethyl)tetrahydro-2H-pyran-2-ylheptadeca-5,7-dienoate from Euclea crispa (L.) Inhibits Ovarian Cancer Cell Growth by Controlling Apoptotic and Metastatic Signaling Mechanisms" was retracted in 2023. Reasons: signs of a paper mill; suspected computer-generated content; unreliable results or conclusions; concerns about the data.

#### 2.6.5. ADME Property Prediction

The selected ligands (isolated compounds) were checked for their ADME properties using QikProp (QikProp, Schrödinger, LLC, New York, NY, 2017). The pharmacokinetics and pharmacodynamics were calculated using the properties of drugs.

### 2.7. Cytotoxicity Analysis

#### 2.7.1. Assessment of Cell Viability

Cell viability was calculated by the MTT assay where the mitochondrial dehydrogenase reduces MTT and forms an insoluble purple formazan [27]. Briefly, the cells (1 × 10^4^/well) were seeded in 96-well plates. The different concentrations of compound were added to the cells (10, 20, 30, 40, 50, and 60 *μ*g/ml) after 24 hours, and the media that contained compound 2 were removed carefully. Then, the cells were washed twice using PBS, and later, 100 ml of medium was added combined with 0.5 mg/ml MTT in PBS to each well. The plates were incubated for 4 h at 37°C and removed, and 200 ml of Tris DMSO was added to each well, placed on a vibrator, and vibrated for about 30 min. The absorbance, which was proportional to cell viability, was subsequently measured at 570 nm in each well using an ELISA Plate Reader (Bio-Rad).

#### 2.7.2. Protein Expression Analysis by Western Blotting

The cell lysates (50 *μ*g) were electrophoresed in 12% sodium dodecyl sulfate-polyacrylamide gel and then transferred onto PVDF membranes. The membranes were incubated with primary antibodies against CXCR4, HER2, Akt, p53, Bcl-2, Bcl-xL, and caspase-9 in Tris-buffered saline (TBS). After washing, the membranes were incubated with HRP-conjugated anti-mouse IgG (1 : 5000) and goat anti-rabbit IgG (1 : 5000). The protein bands were detected using a chemiluminescence system (ECL Kit) and quantified in ChemiDoc XRS Imaging System (Bio-Rad).

### 2.8. Statistical Analysis

The results obtained were expressed as mean ± SD. The statistical comparisons among the groups were performed using the Statistical Package Program (SPSS 10.0).

## 3. Results and Discussion

### 3.1. Isolation and Structural Elucidation of Compound

Plants are bestowed with a variety of phytocompounds, and the phytochemicals present in them are incomparable, and also, they pave way for the discovery of new drugs. Though the synthetic products are available, the demand for therapeutic agents obtained from natural products still ranks at the top since they have fewer or no side effects, and also, the chemical diversity in plants increases the demand for the screening of phytochemicals [28]. There are various chemical compounds present in plants, these compounds are capable of treating certain diseases, and few compounds also possess pharmacological properties such as antioxidant, anticancer, antidiabetic, and anti-inflammatory [12,29]. To identify and isolate, the phytochemicals through chromatographic and spectrometric techniques are employed, and these techniques provide a piece of efficient information regarding the composition of the phytochemicals of plants, especially medicinal plants; it is also extended even to find out the quality and quantity of the compounds extracted from the medicinal plants [30].

The article "(5E,7E)-4,5,6 Trihydroxy-3-(hydroxymethyl)tetrahydro-2H-pyran-2-ylheptadeca-5,7-dienoate from Euclea crispa (L.) Inhibits Ovarian Cancer Cell Growth by Controlling Apoptotic and Metastatic Signaling Mechanisms" was retracted in 2023. Reasons: signs of a paper mill; suspected computer-generated content; unreliable results or conclusions; concerns about the data.

A total of 128 fractions were collected by employing silica gel column chromatography. 320 mg of a single compound (soluble in 95% ethanol) was identified from the fractions 71–82 with the *R*_*f*_ value of 0.41 cm using the TLC analysis (Supplementary Figure 1A), and it indicates that a single compound may be present in a respective fraction. Major absorption bands at *λ*max of 259 nm were observed when a UV-visible spectroscopy analysis (Supplementary Figure 1B) was performed for a single fraction, and at maximum absorbance (0.378), the presence of a single compound was indicated. The FTIR spectrum (Supplementary Figure 2) exhibited characteristic absorption bands for an OH group at 3392, a C=C bond at 1612 cm^−1^, a C=O group at 1714, and the C-H group at 2929, 1462, and 1376 cm^−1^.

However, this study never claimed that those functional groups are present in the proposed chemical compound. The origin of those functional groups is presumably due to impurities present with the chemical compound investigated in the study. Upon extensive purification procedures carried out for the chemical compound, it was noted that the removal of the impurities is very critical (data are not shown) from the interested compound. Meanwhile, we strongly imply that the presence of the impurities did not harm any scientific claims of the manuscript. The ^1^H NMR spectrum (Figure 1) of the compound portrayed an upfield signal at *δ* of 0.85 for terminal methyl groups, a broad singlet at *δ* of 1.28, and a multiplet at *δ* of 1.59 for a long chain of methylene groups and a signal at *δ* of 2.02 for a methylene group linked to the unsaturated group. Furthermore, a pair of multiple signals at *δ* of 5.1 and 5.6 emerged for unsaturated protons. A cluster of signals at *δ* of 4.40, 4.1, 3.90, 3.68, 3.39, and 3.21 reported the presence of a sugar unit. The ^13^C NMR spectrum (Figure 2) of the compound portrayed signals at *δ* of 14.10 for a terminal methyl group, and signals at *δ* of 22.68, 27.95, 27.97, 29.35, 29.65, 29.69, 30.21, 31.440, and 32.81 were due to the long-chain methylene groups. The signals at *δ* of 37.29 and 39.35 were due to the *α*-methylene group carbons to the C=C. Additionally, the signals at *δ* of 61.41, 65.48, and 72.92 suggested the presence of a sugar unit. The signals at *δ* of 114.42, 124.46, 132.17, and 142.81 confirmed the presence of double bonds in the compound. The signal at *δ* of 159.52 depicted the presence of a carbonyl group. Thus, all the above spectral studies revealed that the secluded compound was (5E,7E)-4,5,6 trihydroxy-3-(hydroxymethyl)tetrahydro-2H-pyran-2-ylheptadeca-5,7-dienoate (compound 2) (Figure 3), and the molecular weight is 428.55 g/mol and the molecular formula is C_23_H_40_O_7_, respectively.

The article "(5E,7E)-4,5,6 Trihydroxy-3-(hydroxymethyl)tetrahydro-2H-pyran-2-ylheptadeca-5,7-dienoate from Euclea crispa (L.) Inhibits Ovarian Cancer Cell Growth by Controlling Apoptotic and Metastatic Signaling Mechanisms" was retracted in 2023. Reasons: signs of a paper mill; suspected computer-generated content; unreliable results or conclusions; concerns about the data.

### 3.2. Antioxidant Activity

The antioxidants scavenged the free radicals and act as a defense force of an organism. If the free radicals are not scavenged from the body, they may lead to several other medical complications such as cancer, coronary heart disease, obesity, hypertension, degeneration of brain cells, and nerve cells that lead to spinal muscular atrophy, Huntington's disease, and so on. This investigation recognized the potency of compound 2 to eliminate the free radicals at different concentrations, and this antioxidant activity exhibited by the compound is a remarkable one.

#### 3.2.1. DPPH Radical Scavenging Assay

The standard method used to quantify the potency of antioxidants of plant extracts or elements is DPPH radical scavenging assay. The isolated compound (compound 2) using this technique was observed to have an inhibition at 80% at the highest concentration of 250 *μ*g/ml. Moreover, the IC_50_ value showed that the compounds displayed significant DPPH radical terminating property of 118.97 ± 1.02 *μ*g/ml (Table 1 and Supplementary Figure 3) when analogized with a standard drug of vitamin C (101.94 ± 0.52 *μ*g/ml), and thus, compound 2 could be said to be comparably active with ascorbic acid though vitamin C presented better effect than the compound.

Antioxidants donate a hydrogen atom, and this activity is responsible for the DPPH radical scavenging activity. The DPPH solution turns yellow if a free radical has been scavenged by an antioxidant. The neutralization of the DPPH free radicals is due to the transfer of an electron or hydrogen atom, which in turn leads to the antioxidant activity of plant chemicals [31–33].

#### 3.2.2. Nitric Oxide Radical Scavenging Assay

Sodium nitroprusside when reacted with oxygen forms nitrite and nitric oxide, and this nitric oxide being a ROS indulges in the occurrence of cancer, inflammation, and pathological conditions [34]. Compound 2 inhibits oxygen from forming nitric oxide dependently, and this activity is revealed through this study conducted. The result depicted is shown in Supplementary Figure 4 and Table 1. Compound 2 has an inferior IC_50_ value of 117.79 ± 0.73 *μ*g/mL when compared with a standard drug (107.62 ± 0.12 *μ*g/mL). Inflammatory processes are initiated and proceeded by nitric oxides, and if there is an increase in the level, they poison the tissues, which may lead to vascular damage and other complications. The toxicity increases with the formation of a second reactive compound peroxynitrite anion when a reaction occurs with the superoxide radical. Compound 2 hinders nitrite formation in the process of procreating the radical (N) by direct competition with oxygen. Thus, this study confirms the nitric oxide scavenging activity of compound 2.

The article "(5E,7E)-4,5,6 Trihydroxy-3-(hydroxymethyl)tetrahydro-2H-pyran-2-ylheptadeca-5,7-dienoate from Euclea crispa (L.) Inhibits Ovarian Cancer Cell Growth by Controlling Apoptotic and Metastatic Signaling Mechanisms" was retracted in 2023. Reasons: signs of a paper mill; suspected computer-generated content; unreliable results or conclusions; concerns about the data.

#### 3.2.3. Hydroxyl Radical Scavenging Assay

The inhibitory potential of hydroxyl radical-mediated deoxyribose shown by compound 2 and standard reference in Fe^3+^-EDTA-ascorbic acid and hydrogen peroxide reaction mixture is illustrated in Supplementary Figure 5 and Table 1. The IC_50_ values of compound 2 and ascorbic acids were 98.79 ± 0.39 *μ*g/ml and 93.28 ± 0.19 *μ*g/ml, respectively, and this value reveals an insignificant difference (*p* > 0.05) in the activity of the duo. Lipid peroxidation and various biological damages are caused by major active oxygen species, namely hydroxyl radicals [35]. Above all, going by the presented IC_50_ values, compound 2 could be said to show comparable significant hydroxyl radical scavenging activity with standard ascorbic acid.

#### 3.2.4. Reducing Power Assay

The occurrence of reductones was due to the coupling of reducing agents, and they exhibit an antioxidant action by breaking the free radical chain to donate a hydrogen atom [36]. The di- and mono-hydroxyl substitutions in the aromatic ring have a powerful hydrogen donating capacity, which may render a reducing power for compound 2. The result illustrated in Supplementary Figure 6 revealed that at the highest concentration of 250 *μ*g/ml, the absorbance value of compound 2 had a similar significant reducing power activity (0.78 ± 0.03) with ascorbic acid (0.78 ± 0.06). Higher absorbance is an indication of the strong reducing capacity of the compound and vitamin C.

#### 3.2.5. FRAP Assay

Antioxidants are reducing agents and inactivators of oxidants. They exhibit a reducing property, which serves as a significant indicator of antioxidant activity [37]. The chemical reduction of Fe^3+^ to Fe^2+^ determines the reductive potential of compound 2. The FRAP assay depicted that at 250 *μ*g/ml the maximum absorbance (Supplementary Figure 7) of compound 2 and standard ascorbic acid was 0.82 ± 0.02 and 0.88 ± 0.01, respectively, which are insignificantly different from one another.

The article "(5E,7E)-4,5,6 Trihydroxy-3-(hydroxymethyl)tetrahydro-2H-pyran-2-ylheptadeca-5,7-dienoate from Euclea crispa (L.) Inhibits Ovarian Cancer Cell Growth by Controlling Apoptotic and Metastatic Signaling Mechanisms" was retracted in 2023. Reasons: signs of a paper mill; suspected computer-generated content; unreliable results or conclusions; concerns about the data.

### 3.3. Computational Molecular Analysis

The predominant binding style of a ligand with protein of known 3D structure is predicted using protein-ligand docking. The scores obtained as a result of interactions render suggestions regarding the active site. The binding sites of the proteins guide the docking analysis. To justify the described ligand and protein preparation, the results of the site map molecular docking analysis were taken into account for compound 2 and cyclophosphamide complex [38]. The docking analysis of the secluded element with targeted proteins of HER2 and CXCR4 is shown in Table 2. The HER2-compound 2 complex (Figure 4) has a good Glide score of −7.394 and Glide energy of −51.591 kcal/mol when compared with the HER2-cyclophosphamide complex (Figure 5).

The CXCR4-compound 2 complex (Figure 6) also had a good Glide score of -6.880 and Glide energy of −46.137 kcal/mol when compared with CXCR4-cyclophosphamide complex (Figure 7). In the molecular docking analysis, the isolated compound of compound 2 possesses possible dual inhibitory activity with HER2 and CXCR4 proteins. The ADME property prediction results (Table 3) of secluded natural elements and FDA-approved drug range were satisfactory. Thus, the computational molecular analysis indicates that compound 2 from ethanolic extract of *E. crispa* may possess good anticancer activity.

### 3.4. Effect on Cytotoxicity

Cancer is a life-threatening disease that may even end up to death if not treated at the right time. Ovarian cancer is one of the common benign tumours in female genital organs and has the highest mortality rate of all gynaecological cancer types [39]. Present cancer therapy limitations include the search for new anticancer drugs. The plants constitute an immeasurable source of bioactive compounds for drug discovery. In the MCF-7 human breast cancer cell line, *E. crispa* has been reported to possess an anticancer activity [40]. A study from our laboratories has shown that 29 volatile phytochemicals isolated from the hexane extract of *E. crispa* leaves suggested that these compounds could be an effective drug target for human chemokine receptor (CXCR4) and human epidermal growth factor receptor 2 (HER2) for the growth of an anticancer drug, which was analyzed by molecular docking analysis. Nevertheless, the chemopreventive potential of the plant extract and isolated compound 2 in *in vitro* human cell line model has been reported. Hence, this study analyzed the cytotoxic, antiproliferative, and antiapoptotic potential of the isolated compound 2 in a human ovarian cancer cell line (HO-8910) [6,15]. To assess the cytotoxicity of compound 2 on the increased growth of ovarian cancer cells, HO-8910 cells were treated with different concentrations of the compound (10, 20, 30, 40, 50, and 60 *μ*g) and the cell capability was identified by the MTT method. As depicted in Figure 8, compound 2 exerts its cytotoxicity on ovarian cells and the growth hindrance rate at the concentrations of 30 and 40 *μ*g (*p* < 0.05). Therefore, 30 and 40 *μ*g concentrations were considered for further protein expression analysis. In support of the cytotoxic activity of *E. crispa* that is recorded in this study, the extract had a cytotoxic potential in the human MCF-7 breast cancer cell line (45.7 *μ*g/ml) [40].

The article "(5E,7E)-4,5,6 Trihydroxy-3-(hydroxymethyl)tetrahydro-2H-pyran-2-ylheptadeca-5,7-dienoate from Euclea crispa (L.) Inhibits Ovarian Cancer Cell Growth by Controlling Apoptotic and Metastatic Signaling Mechanisms" was retracted in 2023. Reasons: signs of a paper mill; suspected computer-generated content; unreliable results or conclusions; concerns about the data.

### 3.5. Effect on CXCR4 and HER2 Protein Expression in HO-8910 Cells

Chemokine gradient cells direct cell migration through several processes, both physiological and pathological. Cancer cells show chemokine receptors that react to chemokine-resolving changes in cancer growth and spread [41]. The chemokine receptor 4 (CXCR4) is a G-protein-coupled membrane receptor, expressed by most forms of cancer. CXCR4 performs a pivotal function in the progress of cancer and metastatic spread [42]. It has also been documented that CXCR4-positive is 69% of in situ ductal carcinoma (DCIS) lesions. It has also been suggested that CXCR4 overexpression is of prognostic importance for imaging and diagnostic applications [43]. In our research, the expression of CXCR4 protein in compound 2-treated HO-8910 cells (Figure 9(a)) was found to be significantly reduced (*p* < 0.01) and this analysis agrees with the docking study, indicating that compound 2 modulates the expression of CXCR4 protein in ovarian cancer cells and thus reduces the cell proliferation.

HER2 (ErbB2) belongs to the family of transmembrane tyrosine kinase-type receptors of the epidermal growth factor receptor (EGFR). It contributes to activating its downstream signaling cascades, which could facilitate tumour cell proliferation, metastasis, and angiogenesis [44,45]. The overexpression of this oncogene performs a mandatory function in the growth and progress of cancer cells, and it acts as novel therapeutic target sites for ovarian and breast cancer [6]. In this study, compound treatment to HO-8910 cells expressed a substantial decrease in HER2 protein expression compared with the control cells (Figure 9(b)) and a subsequent substantial reduction (*p* < 0.05) in the Akt protein level (Figure 9(c)), suggesting that compound 2 inhibits chemokines and epidermal growth factor receptor-mediated cell proliferation and metastasis in HO-8910 cells. Hence, the present findings on *in vitro* cell human line and molecular docking analysis indicate that compound 2 from *E. crispa* leaves may serve as a potent CXCR4 and HER2 inhibitor in ovarian cancer treatment.

The article "(5E,7E)-4,5,6 Trihydroxy-3-(hydroxymethyl)tetrahydro-2H-pyran-2-ylheptadeca-5,7-dienoate from Euclea crispa (L.) Inhibits Ovarian Cancer Cell Growth by Controlling Apoptotic and Metastatic Signaling Mechanisms" was retracted in 2023. Reasons: signs of a paper mill; suspected computer-generated content; unreliable results or conclusions; concerns about the data.

### 3.6. Effects on Apoptosis-Related Protein Expression in HO-8910 Cells

The cytotoxic drugs function by activating the intrinsic pathway of apoptosis. Bcl-2 family holds 25 proapoptotic proteins and antiapoptotic members, and these help in balancing the newly generated cells and dying cells. Its subfamily holds proteins that subdue the mechanism of cell death of a few proapoptotic proteins.

The antiapoptotic proteins are expressed more in ovarian cancer. The proteins along with the proapoptotic proteins curb the cell death, thereby increasing the growth of tumour cells, which in turn leads to malignancy [46]. Anti-proapoptotic drugs are used to target the proteins, and this, in turn, inhibits the function of proteins. These drugs stimulate the activation of tumour suppressor protein p53, and this, in turn, reduces antiapoptotic protein expression [47]. In this study, the mechanism observed was similar to that of compound 2 that was treated in the HO-8910 cells. There were a substantial increase (*p* < 0.05) in the expression of proapoptotic protein p53 (Figure 10(a)) and a decrease in the expression of Bcl-2 and Bcl-xL antiapoptotic protein levels (Figures 11(a) and 11(b)). This study clearly states that compound 2 promotes apoptosis through the intrinsic pathway.

The primary apoptosis caspase located in the cytosolic space serves as a mediator. Also, its expression substantially increased in compounds treated HO-8910 cells. Compound 2 in *E. crispa* was postulated to release cytochrome c from the mitochondrial space that unites with the adaptor molecule apoptosis protease-activating factor 1 and inactive caspase initiator, procaspase-9, within the protein complex and forms apoptosome. Through an intrinsic pathway, apoptosis is activated, and the activation is the result of the apoptosome and caspase activation.

## 4. Conclusion

The potential compound (5E,7E)-4,5,6 trihydroxy-3-(hydroxymethyl)tetrahydro-2H-pyran-2-ylheptadeca-5,7-dienoate (compound 2) was secluded and recognized from the ethanolic extract of *E. crispa* leaves using chromatographic and spectroscopic techniques. The antioxidant activity of compound 2 (based on the tested parameters) and its scavenging activities were revealed through the study. *In silico* and *in vitro* studies demonstrate that compound 2 hinders the rapid cell growth in HO-8910 cells by modulating the expression of HER2, CXCR4, and Akt proteins. Also, compound 2 strongly interferes with the apoptotic pathway by inhibiting the growth of ovarian cancer cells. It also downregulated the antiapoptotic proteins and upregulated the protein of the tumour suppressor (p53), paving the way for cell death. The activation of caspase-9 demonstrated that the compound acts through the intrinsic apoptotic pathway. Taken together, this study concludes that compound 2 can serve as a potential antioxidative and chemotherapeutic anticancer agent. Thus, compound 2 can serve as a promising chemotherapeutic anticancer agent for ovarian cancer treatment. Besides, further studies through the *in vivo* model and clinical trials would reveal the nature and expound how potential the drug is in the future.

The article "(5E,7E)-4,5,6 Trihydroxy-3-(hydroxymethyl)tetrahydro-2H-pyran-2-ylheptadeca-5,7-dienoate from Euclea crispa (L.) Inhibits Ovarian Cancer Cell Growth by Controlling Apoptotic and Metastatic Signaling Mechanisms" was retracted in 2023. Reasons: signs of a paper mill; suspected computer-generated content; unreliable results or conclusions; concerns about the data.

## Figures and Tables

**Figure 1:** ^1^H NMR spectrum analysis for compound 2.

**Figure 2:** ^13^C NMR spectrum analysis for compound 2.

**Figure 3:** The structure of (5E,7E)-4,5,6 trihydroxy-3-(hydroxymethyl)tetrahydro-2H-pyran-2-ylheptadeca-5,7-dienoate (compound 2).

**Figure 4:** Docking complex of HER2 with compound 2 generated using Glide XP module of Schrödinger suite is shown in this figure. The proteins, ligand, and binding pockets are represented in ((a) 3D graphics) ribbon, sticks, and surface models, respectively. The residues of the HER2 that are within 4 Å proximities to compound 2 are illustrated in (b) 2D graphics. Dotted lines denote “hydrogen bonds” between the corresponding atoms.

**Figure 5:** Docking complex of HER2 with cyclophosphamide generated using Glide XP module of Schrödinger suite is shown in this figure. The proteins, ligand, and binding pockets are represented in ((a) 3D graphics) ribbon, sticks, and surface models, respectively. The residues of the HER2 that are within 4 Å proximities to the cyclophosphamide are illustrated with (b) 2D graphics. Dotted lines denote “hydrogen bonds” between the corresponding atoms.

**Figure 6:** Docking complex of CXCR4 with compound 2 generated using Glide XP module of Schrödinger suite is shown in this figure. The proteins, ligand, and binding pockets are represented in ((a) 3D graphics) ribbon, sticks, and surface models, respectively. The residues of the CXCR4 that are within 4 Å proximities to compound 2 are illustrated in (b) 2D graphics. Dotted lines denote “hydrogen bonds” between the corresponding atoms.

**Figure 7:** Docking complex of CXCR4 with cyclophosphamide generated using Glide XP module of Schrödinger suite is shown in this figure. The proteins, ligand, and binding pockets are represented in ((a) 3D graphics) ribbon, sticks, and surface models, respectively. The residues of the CXCR4 that are within 4 Å proximities to the cyclophosphamide are illustrated with (b) 2D graphics. Dotted lines denote “hydrogen bonds” between the corresponding atoms.

**Figure 8:** Effect of compound 2 on the viability of ovarian cancer cells. HO-8910 (1 × 10^4^/well) cells were cultured in RPMI 1640 medium supplemented with 10% FBS and incubated with indicated concentrations of compound 2 for 24 h. For cell viability assay, cells were exposed to different doses (0–60 *μ*g/ml) of compound 2 for 24 h, and compound 2 inhibits growth (as determined by MTT assay) of HO-8910 cancer cells. Each bar represents the mean ± SEM of five independent observations and the statistical significance between the control and treated groups at *p* < 0.05 level.

The article "(5E,7E)-4,5,6 Trihydroxy-3-(hydroxymethyl)tetrahydro-2H-pyran-2-ylheptadeca-5,7-dienoate from Euclea crispa (L.) Inhibits Ovarian Cancer Cell Growth by Controlling Apoptotic and Metastatic Signaling Mechanisms" was retracted in 2023. Reasons: signs of a paper mill; suspected computer-generated content; unreliable results or conclusions; concerns about the data.

**Figure 9:** Effect of compound 2 on C-X-C motif chemokine receptor 4 (CXCR 4), human epidermal growth factor receptor 2 (HER2), and Akt protein expression in HO-8910 cells. Cells were treated with 30 and 40 *μ*g of compound for 24 h. The protein levels were quantified using densitometry analysis and are expressed in relative intensity arbitrary unit. Each bar represents mean ± SEM of six independent observations. (a) Compared to control; (b) compared to 30 *μ*g of compound 2.

**Figure 10:** Effect of compound 2 on p53 and caspase-9 protein expression in HO-8910 cells. Cells were treated with 30 and 40 *µ*g of compound for 24 h. The protein levels were quantified using the densitometry analysis and are expressed in relative intensity arbitrary unit. Each bar represents mean ± SEM of six independent observations. (a) Compared to control; (b) compared to 30 *μ*g of compound 2.

**Figure 11:** Effect of compound 2 on antiapoptotic protein (Bcl-2 and Bcl-xL) expression in HO-8910 cells. Cells were treated with 30 and 40 *μ*g of compound for 24 h. The protein levels were quantified using the densitometry analysis and are expressed in relative intensity arbitrary unit. Each bar represents mean ± SEM of six independent observations. (a) Compared to control; (b) compared to 30 *μ*g of compound 2.

**Table 1:** Free radical scavenging capacities of compound 2 from ethanolic extract of *E. crispa* leaves.

Extracts	IC_50_ values (*μ*g/ml)		
	DPPH radical	Nitric oxide radical	Hydroxyl radical
Compound 2	118.97 ± 1.02^a^	117.79 ± 0.73^a^	98.79 ± 0.39^a^
Ascorbic acid	101.94 ± 0.52^b^	107.62 ± 0.12^b^	93.28 ± 0.19^a^

Note: values with different superscript letters on the same row are significantly different from each other at *p* < 0.05.

**Table 2:** Glide scores and Glide energies of CXCR4 and HER2 target proteins and ligands.

S. No.	Compounds	HER2		CXCR4	
		Gscore	GEnergy	Gscore	GEnergy
1	Compound 2	−7.394	−51.591	−6.880	−46.137
2	Cyclophosphamide	−4.621	−32.158	−4.276	−26.992

Note: isolated natural compound and FDA-approved drug complexes are given as calculated from the molecular docking studies.

**Table 3:** ADME property prediction of screened compounds.

S. No.	Compounds	Molecular weight	H-bond donor	H-bond acceptor	Log_*P*_ O/W
1	Compound 2	428.55	5	7	1.7
2	Cyclophosphamide	261.08	1	4	0.6

The article "(5E,7E)-4,5,6 Trihydroxy-3-(hydroxymethyl)tetrahydro-2H-pyran-2-ylheptadeca-5,7-dienoate from Euclea crispa (L.) Inhibits Ovarian Cancer Cell Growth by Controlling Apoptotic and Metastatic Signaling Mechanisms" was retracted in 2023. Reasons: signs of a paper mill; suspected computer-generated content; unreliable results or conclusions; concerns about the data.

## Data Availability

The data used to support the findings of this study are included within the article.

## Supplementary Materials

Supplementary Materials Supplementary Figure 1: (A) single compound identification by the TLC analysis and (B) *λ*max analysis for compound 2 through UV spectrum. Supplementary Figure 2: FTIR spectrum for compound 2, which indicates the presence of functional groups by the characteristic absorptions (1/cm). Supplementary Figure 3: DPPH radical scavenging activity of compound 2. Supplementary Figure 4: nitric oxide radical scavenging activity of compound 2. Supplementary Figure 5: hydroxyl radical scavenging activity of compound 2. Supplementary Figure 6: reducing power activity of compound 2. Supplementary Figure 7: FRAP radical scavenging activity of compound 2. Available at the journal website.
